The article "Greedy Strategies with Multiobjective Optimization for Investment Portfolio Problem Modeling" was published in 2022. Journal: Comput Intell Neurosci.

# Greedy Strategies with Multiobjective Optimization for Investment Portfolio Problem Modeling

**DOI:** 10.1155/2022/4862772

**Published:** 2022-05-19

**Authors:** Xinchen Zhang, Linghao Zhang, Qincheng Zhou, Xu Jin

**Affiliations:** ^1^School of Telecommunications and Information Engineering, Nanjing University of Posts and Telecommunications, Nanjing 210046, China; ^2^School of Science, Nanjing University of Posts and Telecommunications, Nanjing 210046, China

## Abstract

The ultimate purpose of portfolio investment is to reduce investment risk and improve total return on the premise of ensuring reasonable allocation of capital. In this paper, we build a quantitative model to advise on trading based on the price movement of Bitcoin and gold between 2016 and 2021; our goal is to maximize profit while minimizing risk. We mainly use greedy strategies with multiobjective optimization models. For the purpose of obtaining the correct price trend, some popular trend indicator strategies are referred to predict the future price trend in the medium and long term. In addition, we also consider people with different trading preferences and divided them into aggressive, advanced, balanced, and cautious and provided trading strategies for each of these four groups. This gives our model scalability. Finally, we analyze the sensitivity of the model and discuss the impact of trading commission costs on the model results. The model can be applicable to various investment situations.

## 1. Introduction

Investment portfolio refers to a series of assets, such as bonds, stocks, and currency derivatives. Usually, a high-quality investment portfolio should be high liquidity, high stability, high return, low investment risk, etc. Portfolio problem is a kind of very complex decision-making problem. The research on the problem of portfolio is helpful to improve the risk consciousness of decision-makers and can improve the rationality and effectiveness of investment decisions, avoid the blindness of investment, reduce its cost, and improve its return. Under normal circumstances, when investors make decisions, the most concerned issue for investors is to allocate the limited capital effectively and to arrange the order of asset investment reasonably, so as to maximize the overall return and minimize the risk of the portfolio. Investors have different preferences. Risk-averse people want to make investments with as little risk as possible and then they want to make returns; risk-loving people pursue the return on investment, but do not care much about the risks of investment. They believe that high returns can be achieved only by taking high risks. However, even for investors with different attitudes, the ultimate purpose of portfolio investment is to reduce investment risk and improve total return on the premise of ensuring reasonable allocation of capital, so they should still be considered as the most important objective.

As a result of the advanced computer technology, quantitative trading based on modern financial investment theory has become a new hot spot in the development of capital investment market at home and abroad. Rapid response, product diversification, and risk control are the main advantages of quantitative trading. In addition to traditional hedge fund and futures trading, quantitative trading is increasingly being used to trade digital currencies (e.g., Bitcoin). Benefiting from the high volatility of digital currencies, many quantitative strategies have realized excess returns. Generally speaking, we believe that a quantitative strategy is a comprehensive study of market characteristics, market sentiment, and other multifaceted information in order to obtain maximum returns with relatively tolerable risk.

In recent years, the application of machine learning in market forecasting has increased and has basically surpassed the prediction accuracy of traditional time series forecasting models. At the same time, we believe that Bitcoin and gold represent high-risk (up to more than 100 times in five years) and low-risk assets, respectively, and how to consider the dynamic allocation of assets to balance risk and return in trading is a central issue in our article.

In our article, we are required to accomplish the following tasks: (1) Bitcoin and gold spot are selected as a portfolio and we are required to use a quantitative strategy to determine the maximum return at the end of the period for a ternary portfolio (*C*, *B*, *G*) of cash, Bitcoin, and gold. (2) Proving theoptimality of our trading strategy. (3) Analyzing the sensitivity of the model and discussing the impact of trading commission costs on the model results.

## 2. Related Works

### 2.1. Portfolio Optimization Theory

Portfolio optimization theory has been developed for nearly 60 years. Markowitz proposed the return as a random variable and created the mean-variance theory of portfolio selection in 1952, which marks the beginning of quantitative analysis method into the field of financial research [1]. It gradually became the focus of investment research. Konno used a mean-absolute deviation portfolio optimization model in the applications to Tokyo Stock Market [2]. Dellino et al. established a portfolio optimization model using the dynamic target aggregation method [3]. Mercurio et al. used a generalized entropic portfolio optimization (GEPO) [4] and a return-entropy portfolio optimization (REPO) [5] for option portfolio selection. Zhou proposes a multiobjective optimization model for investment portfolio problem and solves it by MOEAs [6]. Gong integrated dynamic risk-tolerance and expected-return levels to develop two coherent fuzzy multiperiod portfolio selection models [7]. Yin's study showed that basing on high-frequency prices data, the realized covariance matrix model can improve the accuracy of the portfolio market risk forecast significantly [8]. Jelena researched the effects of portfolio optimization and especially the Bitcoin investment on portfolio optimization [9]. Taking the risk and return variables into account, we can use different optimization techniques to create an optimal portfolio [10–13], which are aimed to create a balance between risk and return in the financial market.

### 2.2. Greedy Algorithm

Greedy algorithm is characterized for its simpler and faster method to solve some optimization problems, often based on the current situation as the basis of an optimization measure to make the optimal choice, without considering all possible overall situation, saving many time to find the optimal solution to exhaust all possible. It generally follow 4 steps: (1) setting up a mathematical model to describe the problem; (2) dividing the problem into several subproblems; (3) solving each subproblem to obtain the local optimal solution; (4) synthesizing the local optimal solution of the subproblem to get a solution of the original problem. Because greedy algorithms always solve problems from the parts, there is no guarantee that the solution is optimal for the whole. Greedy algorithms have many important applications in *n* traffic offloading, medical service, flexible manufacturing, investment planning, etc. [14–19]. By introducing Chritos's greedy algorithm and the simulated algorithm into PSO, Tang proposed a hybrid particle swarm optimization algorithm with adaptive mulisections to make up for the deficiency of PSO [20]. Based on the greedy strategy, Khuller et al. proposed an approximate algorithm with an approximate ratio of (1 − 1/*e*), although they used the local enumeration method which optimizes the approximate ratio of the algorithm, but the algorithm still has a high time complexity *O*(*n*^(*k*+1)^log  *n*), in solving large-scale BMCP (budgeted maximum coverage problem) cases, but also poor in solving results [21]. Zhang et al. proposed a novel (1 − 1/*e*) approximation method for BMCP with *O*(3*n* [4]) time complexity to improve the speed of this algorithm, but the approximate ratio is not yet improved [22] Ashwin proposed an approximate algorithm A-SUKP based on greedy strategy to solve SUKP, in which the approximate ratio of A-SUKP is 1/(1 − *e*^1/*d*^), where *d* (*d* ≥ 2) is the upper bound on the occurrence of all elements. Obviously, the approximate solution of A-SUKP is unsatisfactory and inefficient as *d* gets larger [23]. Li studied group orthogonal greedy algorithm for change-point estimation of multivariate time series [24].

## 3. Model Preparation

### 3.1. Data

The data used in our model for the empirical application consist only of historical price series for Bitcoin and gold, which were collected between 9/11/2016 and9/10/2021. Gold daily prices (in US dollars per troy ounce) are sourced from the London Bullion Market Association, while Bitcoin daily prices (in US dollars per Bitcoin) are sourced from the Nasdaq Stock Market, take a look at Figures 1 and 2. Bitcoin can be traded every day, so the data are continuous. However, gold has a difference between trading days and nontrading days, and the data are not continuous. We first do a smoothed interpolation of the historical price of gold to facilitate forecasting model (nontrading day scenarios are taken into account in the trading strategy).

### 3.2. Our Research Framework

To simplify the problem, our model does not overly consider low probability events such as global financial crisis, financial systemic risk, natural disasters, and exchange closures, in other words, most of the normal risk is already reflected in the price changes. We consider Bitcoin to be a high risk asset and gold to be low. If we want to get higher returns, we will hold more Bitcoins and give up gold in bitcoin uptrends (under controlled risk). Trend and timing are important propellants to obtain excess returns. We only consider trading on the right side, making trades at the moment of uptrend or trend turn and will not ambush in downtrends.

In this article, considering the background information and restricted conditions identified above, we will use multiobjective optimization to solve this problem. The paper is divided into three main parts for trend trading strategy, multiobjective optimization, and model sensitivity analysis, respectively.

#### 3.2.1. Trend Trading Strategy

We believe that trends are very important. We need to consider the proportion of our portfolio at every moment. A common quantitative strategy is commodity trading advisor strategy, which is called the CTA strategy, a strategy based on price trends. In the trading strategy, we use a LSTM-P neural network model for predicting the values of Bitcoin and gold for the next five days (in this article, we will not discuss LSTM-P neural network model). Then, based on our predicted prices, we combine some trending indicators to identify trading signals. We get the price trend with high probability through trend indicator analysis and use it to classify the trading behaviors into 5 categories.

#### 3.2.2. Portfolio Optimization

We need to consider a return-risk biobjective optimization model. The objective functions are optimized through the expected wealth, the variance, and the conditional value at risk, including transaction costs, investor risk appetite, and investment limits for each asset. Common risk models include mean-variance model and multiobjective evolutionary algorithm. We finally refer to multiobjective model predictive control [25] and Pareto optimization principle to simplify and derive our return-risk model. We obtain the optimal portfolio allocation ratio as the local optimal solution by some constraints obtained by the greedy algorithm.

#### 3.2.3. Model Sensitivity Analysis

After validity and stationarity tests, our article effectively demonstrates the validity and applicability.

## 4. Multiobjective Optimization Control (MOC)

By using the LSTM-P neural network model, we have got the price forecast for the next 5 days from the price data so far, and we have to determine the trading and portfolio ratios together based on the forecast and some other indicators. We believe that both risk and return are required to be considered, so we are going to make a multiobjective optimal control model (MOC) for risk and return.

Before building the MOC model, we introduce some trend technical indicators commonly used in financial quantitative analysis to get the forecast of future price trend. This will be part of the constraints of the multiobjective optimization later.

### 4.1. Trend Prediction Model

We believe that it is not enough to know the forecast data for the next few days. In order to reduce high-frequency trading and lower the error rate, we need to know the change of a price trend in the medium and long-term future (for example, one month).

We refer to 28 technical indicators such as MACD, BOLL, and KDJ. A correlation test was performed (the correlation heatmap is shown in Figure 3).

We finally choose two indicators, MACD and BOLL, to calculate the trend. The former can be briefly explained as the acceleration change of price movement, and the latter can be briefly described as the channel of price movement. The detailed explanation of the indicators is not described here.

Figure 4 shows the MACD and BOLL charts that we plotted for the Bitcoin price. We have only shown a portion of the time to make it look clear.

It is obvious that these two indicators give a good picture of the trend direction of Bitcoin in the medium to long term. We have divided the trend into an uptrend, a downtrend, and an oscillating trend. We obtain the future medium to long-term trend by combining these two indicators and the forecast price for the next 5 days and highlight the resulting uptrend in green (Figure 5).

We assume that it is more cost-effective to buy in uptrends, while buying in downtrends should be eliminated (or positions reduced). This greed-like idea is quantified as constraints to perform multiobjective optimization.

That is, we give the future trend a score *Tr* ∈ (−1,1), indicating the probability of being an uptrend. As a greedy idea, we consider that the species cannot be bought when *Tr* < 0. Here, *Tr* denotes the index of future trend. We have also divided the buy and sell signals corresponding to the gold and Bitcoin trend combinations into 5 categories, which is a constraint and the value of *S* in the risk function CvaR.

Figure 6 shows the buy and sell signals corresponding to the 5 categories of our trend portfolio (green is BTC and yellow is gold).

### 4.2. Multiobjective Optimal Control Model

In order to obtain an optimal portfolio, we need to perform multiobjective dynamic optimization control. In this section, we derive the mathematical principles of the model in detail.

#### 4.2.1. Description of the Model

Multiobjective optimization control (MOC) is used to study the optimization of more than one objective function and satisfies the contradiction between the objectives of multi\objective planning. The model of multiobjective planning consists of two parts: more than two objective functions and several constraints.

In the case described in our problem, our objectives are the maximization of benefits and the minimization of risks. In the following, we will describe the quantitative functions of return and risk, respectively, as well as the constraints on the final set of planning equations.

#### 4.2.2. Returns Calculation

*(1) Basic Variables*. Suppose *η*(*k*) ∈ *ℝ*^2^ is a time series of returns on two risky assets, gold and BTC. *𝔽*=(*F*_*k*_)_*k*≥1_ is a filter on the *σ* domain generated by *η*(*k*) [26]; *a*_1_(*k*) and *a*_2_(*k*) represent the amount of gold and BTC at time *k*, respectively; *η*_1_(*k*), *η*_2_(*k*) represent the returns on gold and BTC at time *k*, respectively. Since we only invest the principal at the beginning, we do not add or withdraw wealth from the portfolio, and the variables *a*_*i*_(*k*), *w*_0_ are all deterministic. Apparently, the value of the assets held at time *k* is

(1) $$\begin{array}{c} W\left(k\right)=a_{1}\left(k\right)+a_{2}\left(k\right). \end{array}$$

In the next instant *k*+1, the value of the assets held is

(2) $$\begin{array}{c} W\left(k+1\right)=\left[1+R_{1}\left(k+1\right)\right]a_{1}\left(k\right)+\left[1+R_{2}\left(k+1\right)\right]a_{2}\left(k\right)\\ =\left[a_{1}\left(k\right)+a_{2}\left(k\right)\right]+\left[R_{1}\left(k+1\right)a_{1}\left(k\right)+R_{2}\left(k+1\right)a_{2}\left(k\right)\right]. \end{array}$$

Then, let the return vector *R*(*k*+1)=(*η*_1_(*k*+1), *η*_2_(*k*+1))^*T*^, *A*(*k*)=(*a*_1_(*k*), *a*_2_(*k*))^*T*^; thus, (10) can be written as

(3) $$\begin{array}{c} W\left(k+1\right)=W\left(k\right)+R^{T}\left(k+1\right)A\left(k\right). \end{array}$$

*(2) Wealth-Variance*. Firstly, some simplifications are made to the model. We consider that the return vector follows the first-order vector autoregressive model VAR(1):

(4) $$\begin{array}{c} \eta \left(k+1\right)=w\left(k+1\right)+A_{1}\eta \left(k\right)+c. \end{array}$$

Here, **A**_1_ is a 2 × 2 coefficient matrix; *c*=(*I*_2_ − *A*_1_)*μ* is a 2 × 1 constant vector, where *μ*=*E*[*η*(*k*)]; *w*(*k*+1) is a 2 × 1 dimensional error vector, and it is Gaussian white noise, that is, *E*[*w*(*k*+1)]=0, *E*[*w*(*k*+1)*w*^*T*^(*k*+1)]=Σ, *E*[*w*(*k*+*i*)*w*^*T*^(*k*+*j*)]=0, *i* ≠ *j*. Thus, based on (12), the expression of the conditional expectation $\bar{\eta }\left(k+m\right)$ is

(5) $$\begin{array}{c} \bar{\eta }\left(k+m\right)=E\left[\eta \left(k+m\right)|F_{k}\right]e\Sigma \\ =E\left[\left(\eta \left(k+i\right)-\bar{\eta }\left(k+i\right)\right){\left(\eta \left(k+j\right)-\bar{\eta }\left(k+j\right)\right)}^{T}|F_{k}\right]\\ =A_{1}^{m}\eta \left(k\right)+\sum_{j=0}^{m-1}cA_{1}^{j}, \end{array}$$

where Σ=∑_*l*=0_^*i*−1^**A**_1_^2*i*−2(*l*+1)^Σ^*w*^=∑_*l*=0_^*i*−1^**A**_1_^2*i*−2(*l*+1)^*E*[*w*(*k*+*l*+1)*w*^*T*^(*k*+*l*+1)] is a 2-order square matrix.

Iterating over (12), one can also calculate the asset value after time *m*.

(6) $$\begin{array}{c} \eta \left(k+m\right)=A_{1}^{m}\eta \left(k\right)+\sum_{j=0}^{m-1}\left[A_{1}^{m-j-1}w\left(k+j+1\right)+A_{1}^{j}c\right]. \end{array}$$

*(3) Conditional Covariance*. To calculate conditional covariance definition,

(7) $$\begin{array}{c} \hat{\eta }\left(k+m\right)=\eta \left(k+m\right)-\bar{\eta }\left(k+m\right)=\sum_{j=0}^{m-1}A_{1}^{m-j-1}w\left(k+j+1\right). \end{array}$$

Then, based on the above definition of the return vector *R*(*k*+*j*), the conditional expectation vector and the conditional covariance vector are defined again here:

(8) $$\begin{array}{c} \bar{R}\left(k+j\right)={\left(\bar{\eta_{1}}\left(k+j\right),\bar{\eta_{2}}\left(k+j\right)\right)}^{T}\bar{R}\left(k+j\right)={\left(\bar{\eta_{1}}\left(k+j\right),\bar{\eta_{2}}\left(k+j\right)\right)}^{T}. \end{array}$$

Thus, $\bar{\Sigma }=E\left[\bar{R}\left(k+i\right){\bar{R}}^{T}\left(k+j\right)|F_{k}\right]=\left[\begin{array}{cc} \Sigma_{2\times 2} & 0_{2\times 1}\\ 0_{1\times 2} & 0 \end{array}\right]$.

According to the above corollary, the expression for the conditional value mean at the moment *k*+*m* becomes obvious:

(9) $$\begin{array}{c} E\left[W\left(k+m\right)|F_{k}\right]=W\left(k\right)+\sum_{j=0}^{m-1}E\left[R^{T}\left(k+j+1\right)|F_{k}\right]A\left(k+j\right). \end{array}$$

#### 4.2.3. Risk Calculation

Assume *X*_*p*_=(*x*_1_, *x*_2_)^*T*^ represents the portfolio of gold and BTC bought or sold now, and set vectors *ξ*=(*ξ*_1_, *ξ*_2_) and $R_{n}=\left(\bar{r_{1}},\bar{r_{2}}\right)$ to represent the vector of returns and the vector of expected returns for the portfolio of gold and BTC, respectively. Here, $\bar{r_{i}}=E\left(\xi_{i}\right)$. Then, the expected value and return of the corresponding portfolio are

(10) $$\begin{array}{c} r_{p}=\sum_{i=1}^{n}x_{i}\xi_{i}=X_{p}\xi ,\\ \bar{r_{p}}=\sum_{i=1}^{n}x_{i}\bar{r_{i}}=X_{p}R_{n}. \end{array}$$

We use CVaR to calculate risk. CVaR is risk evaluation (conditional covariance), also known as the average value of excess losses and the conditional value at risk. It represents the conditional mean value of the maximum loss of an investor's asset portfolio over VaR when investing at a certain confidence level.

Assume *f*(*A*, *R*) is the loss function of the investor's assets, where *a* ∈ *A* ⊂ *ℝ*^*n*^ and *η* ∈ *ℝ*^*n*^. Definition domain *U* denotes the feasible region of the gold and BTC portfolio.

The random vector *R* in the *n*-dimensional vector space denotes the uncertainty variables that have an impact on the loss which the investor cannot capture.

By referring to the relevant literature [26], the CVaR value of an investor's asset portfolio at confidence level *β* and its approximate representation can be expressed as

(11) $$\begin{array}{c} CVaR_{\beta }\left(A\right)=\underset{\alpha \in \mathbb{R}}{\min}F_{\beta }\left(A,\gamma \right), \end{array}$$

where *F*_*β*_(*A*, *γ*) can be approximated as ${\tilde{F}}_{\beta }\left(A,\gamma \right)$:

(12) $$\begin{array}{c} {\tilde{F}}_{\beta }\left(A,\gamma \right)=\gamma +{\left(1-\beta \right)}^{-1}\sum_{s=1}^{S}p_{s}{\left[f\left(A,R_{s}\right)-\gamma \right]}^{+}. \end{array}$$

It can be considered that *S*=5, i.e., there are 5 trend combinations of gold and BTC (refer to Section 4.1). The above is the numerical solution of CVaR value.

Based on the above inversion, we can derive the value equation for multiperiod CVaR, which is used to describe the future risky asset trajectory of multiple investment products.

According to the expression for *η*(*k*+*m*) after *m* instants, one of the trend combinations can be obtained. A new predicted value is obtained by adding a random component to *w*(*k*+*j*+1). For each *j* > 0, at each moment, sample from a normal distribution Σ^*w*^=*E*[*w*(*k*+*l*+1)*w*^*T*^(*k*+*l*+1)] with mean and covariance zero. Then, considering the emergence of S trend combinations, wealth value which is expected becomes a random process:

(13) $$\begin{array}{c} E\left[W\left(k+m\right)|F_{k}\right]=S^{-1}\sum_{s=1}^{S}E\left[W_{S}\left(k+j+1\right)|F_{k}\right]. \end{array}$$

In the same trend combination, the solution of the CVaR value can also be solved:

(14) $$\begin{array}{c} E\left[{\tilde{F}}_{\beta }\left(A,\gamma \right)|F_{k}\right]=\gamma +{\left[\left(1-\beta \right)S\right]}^{-1}\sum_{s=1}^{S}{\left[-E\left[W_{S}\left(k+m\right)|F_{k}\right]-\gamma \right]}^{+}. \end{array}$$

#### 4.2.4. Trading Commission Costs

Trading commissions are proportional costs, which are expressed as a percentage of the transaction amount. Therefore, we should deduct the commission from the expected value, and equations (12) and (14) should be modified as follows (*α* (%) is the commission percentage):

(15) $$\begin{array}{c} E\left[W\left(k+m\right)|F_{k}\right]=W\left(k\right)+\sum_{j=0}^{m-1}E\left[R^{T}\left(k+j+1\right)|F_{k}\right]A\left(k+j\right)\\ -\sum_{j=0}^{m-1}\alpha \left|A\left(k+j\right)-\left(1+E\left[R^{T}\left(k+j\right)|F_{k}\right]\right)A\left(k+j-1\right)\right|,\\ E\left[W\left(k+m\right)|F_{k}\right]=S^{-1}\sum_{s=1}^{S}E\left[W_{S}\left(k+j+1\right)|F_{k}\right]\\ =S^{-1}\sum_{s=1}^{S}\left[W\left(k\right)+\sum_{j=0}^{m-1}E\left[R^{T}\left(k+j+1\right)|F_{k}\right]A\left(k+j\right)\right..\\ -\sum_{j=0}^{m-1}\alpha \left.\left|A\left(k+j\right)-\left(1+E\left[R^{T}\left(k+j\right)|F_{k}\right]\right)A\left(k+j-1\right)\right|\right]. \end{array}$$

#### 4.2.5. Constraints

Investing in gold or BTC has a maximum money limit, which means “you cannot put your eggs in one basket.” Using the greed algorithm, we set different caps for different investment styles. For example, an aggressive investor can allocate more Bitcoins (100% of his or her assets).

Considering the upper limit of the portfolio, i.e., *a*_*i*_^max^(*k*)=*δW*(*k*), *i*=1,2, we can express it as the following constraint:

(16) $$\begin{array}{c} \bar{M}\left(k\right)A\left(k\right)\leq A_{\max}\left(k\right). \end{array}$$

Here, *A*_max_(*k*)=(*a*_max_^*T*^(*k*), ..., *a*_max_^*T*^(*k*+*m* − 1))^*T*^, *A*(*k*)=[*a*^*T*^(*k|k*), ..., *a*^*T*^(*k*+*m* − 1*|k*)]^*T*^, and *a*_max_(*k*)=(*a*_1_^max^(*k*), *a*_2_^max^(*k*)), with *M*=**I**_2_.

Also, the profit obtained from each trading operation must exceed the commission.

(17) $$\begin{array}{c} E\left[W\left(k+m\right)|F_{k}\right]-E\left[W\left(k\right)|F_{k}\right]\\ >\sum_{j=0}^{m-1}\alpha \left|A\left(k+j\right)-\left(1+E\left[R^{T}\left(k+j\right)|F_{k}\right]\right)A\left(k+j-1\right)\right|. \end{array}$$

#### 4.2.6. Multiobjective Optimization

Taking the above inferences into account, the dual objective of “maximum return and minimum risk” is followed in the investment process. Then, the following multiobjective dynamic optimization can be listed based on the constraints mentioned above [26].

(18) $$\begin{array}{c} \underset{U}{\max}E\left[W\left(k+m\right)|F_{k}\right],\\ \underset{U}{\min}E\left[{\tilde{F}}_{\beta }\left(A,\gamma \right)|F_{k}\right]\text{ s.t. }\left\{\begin{array}{c} \bar{M}\left(k\right)A\left(k\right)\leq A_{\max}\left(k\right)\\ E\left[W\left(k+m\right)|F_{k}\right]-E\left[W\left(k\right)|F_{k}\right]>\Delta . \end{array}\right. \end{array}$$

### 4.3. Results of Our Model

We divide the traders into 4 categories: A1 (cautious), A3 (balanced), A4 (advanced), and A5 (aggressive). They have different risk-tolerance (CVaR).

#### 4.3.1. Maximum Return

We first give the results for the aggressive investment style, an investor who places profitability above all factors.

As a result, a maximum return of $ 917,658.45 is obtained with trading commission *α*_*gol*  *d*_=1% and *α*_*BTC*_=2%. Here, *α*_*gol*  *d*_ represents gold commission rate, and *α*_*BTC*_ represents Bitcoin commission rate. The tracking process reveals that this strategy invested all the money (100%) in Bitcoin when it is in an uptrend and gained high returns. The following charts (Figure 7) show the return on total accounts and total assets.

Comparing the chart of Bitcoin, you can see that the return chart of this strategy is highly similar to the trend of Bitcoin's chart. This also shows that the account's main return comes from the volatility of Bitcoin and is a high-risk, high-reward strategy. Conversely, the account has had huge retracements. The data show that the strategy has a maximum retracement of more than 52% in 2019.

#### 4.3.2. Comparison of Different Investment Styles-Pareto Frontier

To determine the optimal control strategy, we use the multiobjective optimization method. In fact, the solution of the multiobjective model is a sequence of control actions called the nondominant or Pareto optimal set.

Mathematically, *J*(*A*(*k*))=[*J*_1_(*A*(*k*)), *J*_2_(*A*(*k*))]^*T*^ is a vector-valued function with 2-objective minimization and if no other feasible sequence of control actions *A*(*k*) exists, the sequence *A*^*q*^(*k*)=(*a*^*q*^(*k*), ..., *a*^*q*^(*k*+*m* − 1)) is called Pareto optimal. A Pareto front is constructed for the problem's solution. The Pareto solutions are given by *P*={*A*^1^(*k*),…, *A*^*S*^(*k*)}, (*S*=5). Thus, we can select the best Pareto solution for the investor. For instance, the investor can tolerate high risk in order to aim for higher returns, or otherwise, he is just conservative and can only accept low risk.  Figure 8 shows the Pareto front charts obtained after the first step of the multiobjective optimization instant.

Figure 9 shows the return curves for the 4 different investment styles with the same trading commissions. Apparently, returns and risks are always proportional.

## 5. Sensitivity Analysis of Our Model

### 5.1. Analysis of the Superiority of Our Model

In fact, our multiobjective (return-risk) model has a higher return under an aggressive investment style if we do not apply predictive data but use real data. Nevertheless, this is already very good, because, after all, we cannot have a god's perspective in real trading.

We also back-test our model against a traditional trend indicator strategy. We have also back-tested the model against a traditional trend indicator strategy. We use a portfolio strategy model based on price forecasting and trend indicators, which is relatively popular in the JoinQuant Quantitative Community, for comparison. The results are shown in Table 1.

In summary, our quantitative strategy has better results than the common strategies.

### 5.2. Analysis of the Impact of Transaction Costs

Based on common sense, we believe that transaction costs are also an important factor in the returns of a strategy. After our model validation, we find that the lower the transaction cost, the higher the strategy return.  Figure 10 shows the impact of different transaction costs on the return curve for aggressive and cautious investment styles.

The data in Figure 10 are obtained when we adjust the commission percentage for Bitcoin and leave the percentage for gold unchanged. This is based on the idea of greed, where getting a bigger return requires investing more Bitcoins, and therefore, the impact of Bitcoin transaction costs on total returns is greater. We control for variables to see the results of running the model, and this is in line with our common sense.

## 6. Conclusions

In this paper, we build a quantitative model to advise on trading based on the price movement of Bitcoin and gold between 2016 and 2021. We mainly use greedy strategies with multiobjective optimization to balance risk and return in trading. Such model end up with a maximum ending return of 91765.85% (aggressive) for this portfolio after 5 years of quantitative trading, with an annualized return of 291.32% and ending assets of $ 917,658.45 (opening assets are $1,000).

The strengths of our work are as follows: (1) to obtain the price trends in the medium and long term, we integrate some common trend indicators with the predicted prices to further improve the correctness of the obtained price trends. (2) Combining greedy strategies with multiobjective optimization to minimize risk and maximize return. (3) Pareto frontier is provided for investors with different preferences. (4) The model can be applicable to various investment situations (*Note.* The model is universal because the portfolios in multiobjective optimization in Section 4 can be extended to N, which only requires adding dimensionality to some vectors and matrices.)

The weaknesses of our work are as follows: (1) the model is not well trained, as only 5 years of price data are used. (2) We filter out the high-frequency price fluctuations in the short term and only considered the medium and long-term price trends, thus reducing the returns to some extent. (3) Some of the models simply use greedy algorithms, which only consider the possible local optimal solutions, but not necessarily the overall optimal solutions.

In short, although our model has a considerable degree of applicability and extremely promising returns, the investment industry is ever-changing and no model can predict all situations and suggest the perfect trading scenario. One needs to be very careful when entering the investment industry and must be well prepared. As Warren Buffett said, “Obviously, every investor will make mistakes. A reasonably intelligent, informed, and diligent person can judge investment risks with a useful degree of accuracy.” If you cannot control your emotions and are easily tempted by price fluctuations, then leave the trading to the computer! The future of financial markets will be a battleground between quantitative trading strategies based on objective data analysis and forecasting.

## Figures and Tables

**Figure 1:** Gold daily price.

**Figure 2:** BTC daily price.

**Figure 3:** Correlation heatmap of indicators.

**Figure 4:** Charts of BOLL/MACD of Bitcoin price (2020-10 to 2021-05).

**Figure 5:** Charts of Bitcoin price uptrend period (2020-10 to 2021-05).

**Figure 6:** Trading operation chart under 5 trend combinations.

**Figure 7:** Total account investment income chart.

**Figure 8:** Pareto front returns, CVaR.

**Figure 9:** Return curves of four different investment styles.

**Figure 10:** Impact of different transaction costs.

**Table 1:** Statistical characteristics of the data before and after processing.

Comparison parameters	Our model	Other model
Number of trades	133	235
Back-test time (same platform)	126.5s	62.7s
Percentage of profitable operations	79.43%	55.56%
Total yield	91765.85%	1940.15%
Max. continuous retracement	15.78%	29.7%

## Data Availability

The dataset used to support the findings of this study are available from the corresponding author upon request.
